# Biogenic Silver Nanoparticles of *Clinacanthus nutans* as Antioxidant with Antimicrobial and Cytotoxic Effects

**DOI:** 10.1155/2021/9920890

**Published:** 2021-05-13

**Authors:** Hock Ing Chiu, Che Nurul Azieyan Che Mood, Nur Nadhirah Mohamad Zain, Muggundha Raoov Ramachandran, Noorfatimah Yahaya, Nik Nur Syazni Nik Mohamed Kamal, Wai Hau Tung, Yoke Keong Yong, Chee Keong Lee, Vuanghao Lim

**Affiliations:** ^1^Integrative Medicine Cluster, Advanced Medical and Dental Institute, Universiti Sains Malaysia, Bertam, 13200 Kepala Batas, Penang, Malaysia; ^2^Department of Chemistry, Faculty of Science, Universiti Malaya, Kuala Lumpur 50603, Malaysia; ^3^School of Pharmacy, University of Nottingham Malaysia, Jalan Broga, Semenyih 43500, Malaysia; ^4^Department of Human Anatomy, Faculty of Medicine and Health Sciences, Universiti Putra Malaysia, 43400 Serdang, Selangor, Malaysia; ^5^Bioprocess Technology Division, School of Industrial Technology, Universiti Sains Malaysia, Gelugor, 11800 Penang, Malaysia

## Abstract

Silver nanoparticles (AgNPs) previously synthesised using leaf (AgNP-L) and stem (AgNP-S) extracts of *Clinacanthus nutans* (*C. nutans*) were tested to evaluate antimicrobial, antioxidant, and cytotoxicity activities. The AgNPs showed good inhibition against bacteria, but not fungi. The inhibition results showed the highest activity against *Staphylococcus aureus* (*S. aureus*) with 11.35 mm (AgNP-L) and 11.52 mm (AgNP-S), while the lowest inhibition was against *Escherichia coli* (*E. coli*) with 9.22 mm (AgNP-L) and 9.25 mm (AgNP-S) in the disc diffusion method. The same trend of results was noted in the well diffusion method. The IC_50_ of AgNP-L and AgNP-S in 2,2-diphenyl-1-picrylhydrazyl (DPPH) and 2,2′-azino-bis (3-ethylbenzothiazoline-6-sulfonic acid) (ABTS) assays was 417.05 *μ*g/mL and 434.60 *μ*g/mL, as well as 304.31 *μ*g/mL and 326.83 *μ*g/mL, respectively. Ferric reducing power (FRAP) assay showed that AgNP-L [872.389 *μ*mol/L Fe(II)] and AgNP-S [612.770 *μ*mol/L Fe(II)] exhibited significantly (*p* < 0.05) greater antioxidant activities than leaf extract (CNL) [152.260 *μ*mol/L Fe(II)] and stem extract (CNS) [110.445 *μ*mol/L Fe(II)] of *C. nutans*. The AgNPs were also proven to possess cytotoxic effects on the breast (MCF-7), cervical (HeLa), and colon (HT-29) cancer cells in a dose-dependent manner. AgNP-S and AgNP-L showed significantly (*p* < 0.05) higher cytotoxicity against MCF-7 (117.43 *μ*g/mL) and HT-29 (78.47 *μ*g/mL), respectively. In conclusion, the biosynthesised AgNPs from aqueous extract leaves and stem of *C. nutans* have demonstrated promising potential towards antioxidant, antimicrobial, and cytotoxicity activities.

## 1. Introduction

AgNPs are well known as effective antimicrobial agents against bacteria and fungi [1–4]. Therefore, they have been studied in bacterial applications, for instance, in the medical, cosmetics, food, and textile industries [5–8]. Various skin diseases caused by pathogenic microorganisms are treated with antibiotics. Commonly prescribed antibiotics include erythromycin, clindamycin, tetracycline, penicillin, and ciprofloxacin [9]. Due to the development of antibiotic resistance, researchers are keen to identify alternatives in the development of new antibacterial agents. The biosynthesis of AgNPs can overcome antibiotic resistance and reduce costs compared to conventional antibiotics [10].

Side effects have been observed in synthetic antioxidants such as butylated hydroxytoluene (BHT) and hydroxyanisole (BHA). Low doses of tested BHA appear to be toxic to Vero cells with mitochondrial function loss based on an MTT assay [11]. Several studies reported significant antioxidant activity of the *C. nutans* extract [12, 13]. Thus, the biocompatible *C. nutans*-derived AgNPs could be an alternative for synthetic antioxidants. AgNPs demonstrated inhibition of free radicals, such as reactive oxygen species (ROS) produced from metabolic reactions to prevent damage to tissues or cells [14, 15]. A previous study reported that the synthesised AgNPs using *Costus afer* aqueous leaf extract showed higher antioxidant activity compared to the leaf extract only [16]. AgNPs may, therefore, be a new/novel antioxidant agent with the ability to avoid side effects exhibited by synthetic antioxidants.

In addition to antibacterial and antioxidant properties, the plant-derived AgNPs are widely studied for their cytotoxic effects against cancer cells [17]. Cancer cells are formed from the transformation of normal cells over a number of stages. These could be based on interactions between genetics and external influences, such as physical, chemical, and biological carcinogens [18]. Drug resistance can occur even after chemotherapy treatment [19]. Therefore, alternative biocompatible and cost-effective chemotherapy drugs are needed. It is evident that plant-derived AgNPs have the potential to inhibit the proliferation of cancer cells [20, 21]. Additionally, cytotoxicity of AgNPs has been reported to induce apoptosis of cancer cells through mitochondrial damage and oxidative stress leading to cell death [22, 23]. The aim of this project is, therefore, to assess the antimicrobial, antioxidant, and cytotoxicity properties of *C. nutans*-derived AgNPs that were previously synthesised [13].

## 2. Materials and Methods

### 2.1. Materials

Glacial acetic acid, methanol, and sodium acetate were purchased from QReC, Selangor, Malaysia. DPPH, 2,4,6-tris(2-pyridyl)-1,3,5-triazine (TPTZ), ABTS reagent, 3-(4,5-dimethylthiazol-2-yl)-2,5-diphenyltetrazolium bromide (MTT) reagent, iron(II) sulphate (FeSO_4_.7H_2_O), and BHA were obtained from Sigma-Aldrich, Missouri, USA. Mueller Hinton Agar (MHA), Mueller Hinton Broth (MHB), Potato Dextrose Broth (PDB), Sabouraud Dextrose Agar (SDA), and commercial silver nanoparticles (C-AgNP) were acquired from Merck, Darmstadt, Germany. Gentamycin sulphate, nystatin, and hydrochloric acid (HCl) were provided by Biobasic, Ontario, Canada. Glycerol was obtained from System®, Selangor, Malaysia. Potassium persulphate was purchased from Acros Organics, New Jersey, USA. 0.25% Trypsin-EDTA, RPMI 1640, penicillin-streptomycin, foetal bovine serum (FBS), L-glutamine, and Dulbecco's Modified Eagle Medium (DMEM) were acquired from Gibco®, New York, USA. 5-fluorouracil (5-FU) was purchased from Tokyo Chemical Industry, Tokyo, Japan. 3-(4,5-dimethylthiazol-2-yl)-5-(3-carboxymethoxyphenyl)-2-(4-sulfophenyl)-2H-tetrazolium (MTS) kit was provided by Promega, WI, USA. Phosphate buffer saline (PBS) was obtained from Invitrogen, New York, USA.

### 2.2. Synthesis of AgNPs

Synthesis of AgNP-S and AgNP-L from CNS and CNL, respectively, was conducted according to our previous published work [13].

### 2.3. Antimicrobial Activities of Synthesised AgNPs

The antimicrobial activities were tested using the disc and well diffusion methods in the presence of an inhibition region. Then, the broth-microdilution approach was used to achieve the minimum inhibitory concentration (MIC) and minimum bactericidal concentration (MBC).

#### 2.3.1. Microorganisms

The antimicrobial activities were tested against Gram-negative bacteria: (1) ATCC 27853 *Pseudomonas aeruginosa* (*P. aeruginosa*) and (2) ATCC 25922 *E. coli*; Gram-positive bacteria: (1) ATCC 25923 *S. aureus*, (2) ATCC 12228 *Staphylococcus epidermidis* (*S. epidermidis*), and (3) ATCC 19615 *Streptococcus pyogenes* (*S. pyogenes*); and fungi: (1) CA 1395 *Candida albicans* (*C. albicans*) and (2) *Candida glabrata* (*C. glabrata*). The bacteria and fungi were obtained from the Microbiology Laboratory of Clinical Trial Complex, Advanced Medical and Dental Institute (AMDI), USM, and Infectomics Cluster, AMDI, USM, respectively. The strains were stored in 10% glycerol at −80°C until further use.

#### 2.3.2. Preparation of Media

MHA was used for bacterial cultures. The MHA was autoclaved at 121°C for 15 min. Then, the media were poured into a sterile Petri dish (Bio-Rad, California, USA), and it was left to solidify for 24 h at room temperature to avoid contamination. The same protocol was applied for fungi with SDA as the media. The plates were labelled and stored at 4°C in a sealed plastic bag till further need and prewarmed in an incubator at 37°C prior to the experiment.

#### 2.3.3. Preparation of Inoculum and Samples

A single colony was transferred from the stock culture to 10 mL of MHB and PDB for bacteria and fungi, respectively. The culture suspension was incubated at 37°C for 24 h. Dilution of the culture with either MHB or PDB was performed corresponding to 1-2 × 10^8^ CFU/mL of the 0.5 McFarland's standard using a UV-VIS spectrophotometer and measured at 600 nm. The absorbance should be at 0.1 equivalent to 10^8^ CFU/mL concentration. Each sample (5 mg) was dissolved in 1 mL of distilled water (dH_2_O). A sonicator (WUC-A10H, Wise Clean, Sonic Wise, California, USA) was used to sonicate the samples for 15 min. Then, the samples were sterile filtered before further use.

#### 2.3.4. Disc Diffusion Method

The procedure was carried out according to the Clinical and Laboratory Standards Institute (CLSI) (M02-A11). Briefly, the prepared inoculum solution was swabbed onto MHA and SDA with a sterile cotton swab. Next, sterile Whatman filter paper (6 mm) (Maidstone, UK) was added with 20 *μ*L of tested samples. The positive controls were gentamicin and nystatin. The discs were gently pressed on the agar and incubated with bacteria and fungi at 37°C and 30°C for 24 and 48 h, respectively. A clear inhibition zone was measured and expressed in millimetre (mm).

#### 2.3.5. Well Diffusion Method

A well of 6 mm in diameter was punctured using sterile pipette tips. Then, the inoculum solution was swabbed on the agar with a sterile cotton swab. Next, 20 *μ*L of the sample was added to each well. The positive controls were gentamicin and nystatin. On the other hand, the negative control was dH_2_O. Diffusion of samples into the agar was conducted for 1 h. Then, bacteria were incubated on the plate at 37°C and fungi at 30°C. The inhibition zones were obtained after 24 h for bacteria and 48 h for fungi [24].

#### 2.3.6. Broth-Microdilution Assay

A broth-microdilution assay was utilised to assess the MIC and MBC. The method described by the Clinical and Laboratory Standards Institute (CLSI) (M07-A9) was used, with certain modifications. A serial dilution (7.8125 *μ*g/mL to 1000 *μ*g/mL) of the sample was prepared in 96-well plates flat bottom. Each well contained a sample (20 *μ*L) and inoculum suspension (180 *μ*L). The positive and negative controls were gentamicin and dH_2_O, respectively. The plate was incubated at 37°C for 24 h. Every well was pipetted with MTT in PBS solution (50 *μ*L, 0.5 mg/mL) after the incubation time. After that, the plate was incubated for 30 min. The appearance of a dark purple colour indicated the presence of live bacteria. To determine the MBC values, 10 *μ*L from the wells without purple colour were streaked on MHA and incubated at 37°C for 24 h. After 24 h, the MBC was assessed to differentiate between bactericidal (no growth of bacteria on the plate) and bacteriostatic (bacteria growth on the plate) agents from the samples [25].

### 2.4. Antioxidant Activities

The antioxidant activities were determined using the DPPH, ABTS, and FRAP assays. Serial dilutions of twofold were performed (31.25, 62.5, 125, 250, and 500 *μ*g/mL) for each sample from their stock solution (1000 *μ*g/mL).

#### 2.4.1. DPPH Radical Scavenging Assay

The radical scavenging DPPH method of antioxidant activity was adapted with some modifications from [26, 27]. Briefly, in a 96-well plate, samples (50 *μ*L) and 0.2 mM DPPH in methanol (150 *μ*L) were added. The plate was incubated for 30 min in the dark, and the absorbance was then measured at 517 nm with microplate readers. The calculation of the antioxidant activity was based on

(1) $$\begin{array}{c} \text{DPPH radical scavenging }\left(\text{\%}\right)=\frac{{\text{Ab}}_{\text{control}}-{\text{Ab}}_{\text{sample}}}{{\text{Ab}}_{\text{control}}}\times 100, \end{array}$$

where Ab_control_ is the DPPH solution absorbance while Ab_sample_ is the DPPH solution with sample absorbance.

#### 2.4.2. ABTS Radical Scavenging Assay

With some modifications, the ABTS radical scavenging assay was adapted from [28]. Briefly, the working solution of ABTS cation radical was prepared by mixing 7 mM ABTS solution and 2.45 mM potassium persulphate at 1 : 1 ratio, and this was kept at room temperature for 16 h in the dark. The working solution was diluted with ethanol, and the absorbance at 734 nm was measured using a microplate reader. Each well was pipetted with the sample (20 *μ*L) and ABTS working solution (180 *μ*L). In the dark, this mixture was incubated for 6 min at room temperature, and the absorbance was measured at a wavelength of 734 nm. As the positive control, the sample was compared with BHA. The ABTS radical scavenging calculation was based on

(2) $$\begin{array}{c} \text{ABTS radical scavenging}\left(\%\right)=\frac{{\text{OD}}_{\text{control}}-{\text{OD}}_{\text{sample}}}{{\text{OD}}_{\text{control}}}\times 100, \end{array}$$

where the absorbance of ABTS working reagent with ethanol is OD_control_ and the absorbance of ABTS working reagent with the sample is OD_sample_.

#### 2.4.3. FRAP Assay

With some changes, the FRAP test was modified according to [29]. In brief, the acetate buffer (0.3 M, pH 3.6) was prepared by mixing 46.3 mL of sodium acetate (0.3 M), 3.7 mL of acetic acid (0.3 M), and 50 mL of dH_2_O. Then, a mixture of 0.010 M TPTZ solution in 0.040 M HCl, 0.020 M FeCl_3_, and acetate buffer in the proportion of 1 : 1 : 10 (v/v/v) was prepared for FRAP reagent. The test was performed using a 96-well plate, and 20 *μ*L of samples was mixed in the dark at an ambient temperature with 180 *μ*L FRAP reagent. After 30 min, the absorbance of the sample was measured at 593 nm using a microplate reader. The FeSO_4_.7H_2_O standard curve was constructed in the range of 31.25 to 2000 *μ*mol/L, and the FRAP activity was calculated in *μ*mol of ferrous equivalent per *μ*g dry extract (*μ*mol Fe(II)/*μ*g sample).

### 2.5. Cytotoxicity Studies

The cytotoxicity tests against MCF-7, HT-29, and HeLa cancer cell lines were carried out on the basis of their percentage of viability after treatment.

#### 2.5.1. Cell Lines and Culture Media

The cell lines HT-29, HeLa, and MCF-7 were obtained from the American Type Culture Collection (ATCC). In DMEM, HeLa cell lines were maintained, while HT-29 and MCF-7 were maintained in RPMI 1640. 1% (v/v) L-glutamine, 10% (v/v) FBS, and 1% (v/v) penicillin-streptomycin were applied to both media at 37°C in the carbon dioxide (CO_2_) incubator (Heraeus BB15, Thermo Scientific, Massachusetts, USA).

#### 2.5.2. Preparation of Cell Concentration and Subculture

The cells were used upon reaching 80% confluent. The old media were pipetted out and rinsed with 5 mL of PBS. Then, 0.5 mL of 0.25% Trypsin-EDTA was applied and incubated in a CO_2_ incubator for 3 min. A 15 mL centrifuge tube was used to contain the solution. 5 mL of fresh media was then applied, and the mixture was centrifuged for 5 min at 1000 rpm (Heraeus Megafuge 16, Thermo Scientific, Massachusetts, USA). The supernatant was removed, and the pellets in 1 mL of complete media were resuspended. 50 *μ*L of suspension was added to 50 *μ*L of Trypan Blue and placed into a slide counter using an automated cell counter TC10 (Bio-Rad, Richmond, California) to count the total cells. At concentrations of 1 × 10^4^ cells/well (HT-29), 5 ×  10^3^ cells/well (MCF-7), and 1 × 10^4^ cells/well (HeLa), the cells were seeded. The residual suspension was subcultured into a new flask and incubated for further use at 37°C in a CO_2_ incubator.

#### 2.5.3. Cell Viability Using MTS Assay

In a 96-well plate, HT-29 (1 × 10^4^ cells/well), MCF-7 (5 × 10^3^ cells/well), and HeLa (1 × 10^4^ cells/well) were seeded. The old media were pipetted out after 24 h and replaced with sample-containing media (12.5, 25, 50, 100, and 200 *μ*g/mL). The untreated cells were used as control. The samples used were AgNP-L, AgNP-S, CNL, CNS, C-AgNP, and 5-Fu as the positive control. Then, after 72 h of incubation time, an MTS reagent (20 *μ*L) was added to each well. The plates were then incubated for a further 4 h in the CO_2_ incubator again. A microplate reader was used to measure the absorbance at 490 nm. The cell viability (%) was calculated using

(3) $$\begin{array}{c} \text{Cell viability }\left(\%\right)=\frac{{\text{OD}}_{\text{sample}}\;}{{\text{OD}}_{\text{control}}}\times 100, \end{array}$$

where OD_sample_ is the sample absorbance of the treated cells, and OD_control_ is the absorbance of the untreated cells.

### 2.6. Statistical Analysis

All of the above experiments were conducted in triplicate and expressed as mean ± standard deviation (SD). One-way variance analysis (ANOVA) and Tukey's honest significant difference (HSD)/Dunnett's *t*-test were used for the statistical analysis. The difference was considered statistically significant if *p* < 0.05.

## 3. Results and Discussion

### 3.1. Antimicrobial Activities

Gram-positive bacteria [*Staphylococcus epidermidis* (SE), *Staphylococcus aureus* (SA), and *Streptococcus pyogenes* (SE)], Gram-negative bacteria [*Pseudomonas aeruginosa* (PA) and *Escherichia coli* (EC)], and fungi [*Candida glabrata* (CG) and *Candida albicans* (CA)] were used to assess the antimicrobial activity of AgNPs. To screen for the presence of antimicrobial activity, the disc and well diffusion method was conducted. The microdilution of the broth was then carried out to obtain the values of MIC and MBC. *Staphylococcus* and *Streptococcus* are common bacteria genera present on the human skin [30], while *S. epidermidis*, *S. aureus,* and *P. aeruginosa* are among the normal “resident” bacteria on human skin. Skin disease can occur when the resident microorganism transforms into pathogenic forms under certain conditions [31, 32]. *S. aureus* is one of the main pathogenic bacteria which can cause various illnesses from minor skin infections to life-threatening diseases. *P. aeruginosa* can lead to dermatitis and even deeper soft-tissue infections [33]. *C. albicans* is the most virulent among other *Candida* species [34].

The inhibition zones of the AgNPs against pathogenic microorganisms are shown in Tables 1 and 2. The concentrations used in the experiments were fixed for all samples at 1000 *μ*g/mL.  Table 1 summarises the antimicrobial activity against microorganisms using the disc diffusion method. Samples AgNP-L and AgNP-S showed antimicrobial activity compared to plant extracts as there was a presence of inhibition zones after 24 h of incubation. Based on the results of the disc diffusion method, AgNP-L and AgNP-S showed the highest activities against *S. aureus* with 11.35 mm and 11.52 mm, respectively. However, both AgNPs demonstrated the lowest activity levels against *E. coli* with inhibition zones at 9.22 mm (AgNP-L) and 9.25 mm (AgNP-S). The inhibition zones of AgNPs (AgNP-L and AgNP-S) were significantly higher than the plant extracts (CNL and CNS). Interestingly, both AgNPs showed the highest activity against *S. aureus* with inhibition zones of 18.29 mm (AgNP-L) and 17.24 mm (AgNP-S) in the well diffusion method (Table 2). Coincidentally, both also displayed the lowest activity against *E. coli* with inhibition zones of 12.83 mm and 13.41 mm, respectively. There were no inhibition zones noted in samples using the aqueous plant extract (CNL and CNS). Despite showing higher antimicrobial activity against the pathogenic microorganisms, the AgNPs showed significant antimicrobial activity inhibiting the growth of the pathogenic microorganisms. However, no activity was observed when AgNPs and plant extracts were tested on fungi (*C. albicans* and *C. glabrata*).

#### 3.1.1. Broth-Microdilution Assay

Based on the antimicrobial activity using disc and well diffusion methods, the samples that produced inhibition zones (AgNP-L, AgNP-S, and gentamicin) were further used for the broth-microdilution assay to determine the MIC and the MBC. Based on the result of MBC, the bactericidal and bacteriostatic properties of the samples against pathogenic microorganisms can be determined. Bactericidal refers to the ability to kill microorganisms while bacteriostatic agents are able to inhibit microorganisms. Plates with no growth of bacteria indicate bactericidal properties while plates with bacteria growth indicate bacteriostatic abilities [25].  Table 3 shows the MIC and MBC values for the AgNPs. To determine the antimicrobial activity, the disc diffusion method was used because it is a simple and reliable method with a minimum cost [35]. However, MIC could not be determined because it requires a large range of concentrations and is not economic compared to disc or well diffusion. Therefore, to determine the MIC values, a broth-microdilution assay was carried out.

The MIC was performed in a 96-well plate and incubated at 37°C for 24 hours. The MTT reagent was used as an indicator after 24 h. The change in colour from purple to yellow was indicative of bacteria death [25]. The MIC of AgNP-L was reported at the concentration of 250 g/mL against *S. aureus*, *S. epidermidis*, *S. pyogenes*, and *P. aeruginosa*, and it was reported at 125 *μ*g/mL against *E. coli*. As for *S. aureus*, *S. epidermidis*, and *S. pyogenes*, the MIC of AgNP-S was reported at the concentration of 250 *μ*g/mL, and it was reported at 125 *μ*g/mL for *E. coli* and *P. aeruginosa*. The AgNP-L MBC was the same as the bactericidal MIC due to the absence of bacterial growth at 250 *μ*g/mL against *S. aureus*, *S. epidermidis*, *S. pyogenes*, and *P. aeruginosa*, and it was reported at 125 *μ*g/mL against *E. coli*. In MIC, the MBC of AgNP-S also demonstrated the same concentration. There were no MIC and MBC for fungi because there were no inhibition zones using the disc or well diffusion methods.

From the results in Tables 1 and 2, AgNP-L and AgNP-S showed inhibition zones compared to plant extracts (CNL and CNS). Plant extracts at 1000 *μ*g/mL showed no inhibition zones. Previous studies have investigated the antimicrobial activity of *C. nutans.* However, results showed insignificant activity against acne-inducing bacteria even at high concentrations (5 mg/mL) [36]. The *C. nutans* leaf extract showed important antimicrobial effects against *E. coli* and *S. aureus*, with MIC values of 12.5 mg/mL [37].

As for AgNPs, the result in Tables 1 and 2 suggests that Gram-positive bacteria possess better inhibition zones compared to Gram-negative bacteria. Similar results were found by [38] where *S. aureus* inhibited a higher zone than *E. coli*, thus suggesting the absorption and accumulation of AgNPs on the cell wall. Nevertheless, insignificant inhibition zones occurred against *C. albicans* and *C. glabrata*. In the AgNPs synthesis with *Lantana camara* L. leaves, Gram-positive (*S. aureus*; 28 mm) bacteria have a larger inhibition zone than Gram-negative bacteria (*P. aeruginosa*, 21 mm; and *E. coli*, 22 mm) using the well diffusion method.

The other mechanism is due to the size of AgNPs. The small size of AgNPs results in a large surface area to volume ratio, and this is important in antimicrobial activity against pathogenic bacteria. AgNPs are able to easily attach and penetrate the microorganisms compared to bigger particles [10]. In a comparative study, size-controlled AgNPs with 5 nm showed the lowest minimum inhibitory concentrations compared to 100 nm against *E.coli, B. subtilis*, and *S. aureus* [39].

A former study hypothesised that cell death is caused by high concentrations of positive potassium (K^+^) ions in the extracellular fluids as a consequence of bacterial cell damage by AgNPs [40]. The study also reported that the amount of proteins released by the bacterial cells increased with the concentration of AgNPs. Another study reported that silver ions interrupt the enzymes and proteins needed for adenosine triphosphate (ATP) production, thus disturbing the life cycle of the cell and leading to cell death [41]. On the other hand, a study by [42] reported that cell death could occur due to the interaction of silver with protein. AgNPs react with sulphur-containing amino acids with the abundance of sulphur-containing proteins within and outside the bacterial cell, thus influencing the viability of the bacterial cell. Furthermore, silver ions from the nanoparticles interact with phosphorus in deoxyribonucleic acid (DNA), resulting in the inactivation of DNA replication and the inhibition of enzyme functions [43, 44]. Transmission electron microscopy (TEM) analysis showed a big gap between the cytoplasm and cell wall of the *E. coli* after treatment with silver, thus confirming the presence of phosphorous as a primary component in DNA molecules [45].

### 3.2. Antioxidant Activities

Reactive oxygen species (ROS) released in excess during metabolic reactions in the human body cause cell damage [46]. ROS can cause the development of cancer, cardiovascular disease, inflammation, aging, and neurological diseases [47]. Antioxidants function as scavengers to the free radicals caused by ROS, which decreases the risk of chronic disease [48]. Antioxidant activity of AgNPs was analysed in serial concentrations of 31.25, 62.5, 125, 250, and 500 *μ*g/mL using DPPH, ABTS, and FRAP assays. These three assays were chosen as they are simple and inexpensive and produce fast results.

#### 3.2.1. DPPH, ABTS, and FRAP Assays

Figure 1(a) shows the effects of radical scavenging activity for CNL, CNS, C-AgNP, AgNP-L, and AgNP-S compared with the standard antioxidant BHA. Inhibitory activity against the DPPH radical was seen in the samples examined. The determined half-maximal inhibitory concentration (IC_50_) values for CNL and CNS were >500 *μ*g/mL, 417.05 *μ*g/mL (AgNP-L), 434.60 *μ*g/mL (AgNP-S), and 40.97 *μ*g/mL (BHA). The results showed that control (BHA) exhibited significantly higher values, while C-AgNP showed significantly lower IC_50_ values than CNL, CNS, AgNP-L, and AgNP-S. Based on the order of BHA > AgNP-L > AgNP-S > CNL > CNS > C-AgNP, the scavenging effects of samples on radical DPPH decreased.

It was discovered that each sample's capacity to scavenge free radicals differed and increased in a dose-dependent manner. Therefore, the interaction between sample form and concentration had significantly affected CNL, CNS, C-AgNP, and control (BHA). There were no significant differences between CNL and CNS for all concentrations. The same goes for AgNP-L and AgNP-S. However, there was a significant difference between the plant extracts (CNL and CNS) and AgNPs (AgNP-L and AgNP-S). Both AgNPs were significantly higher compared to C-AgNP. It shows that AgNPs are more effective as antioxidant agents compared to *C. nutans* plant extracts at all concentrations.

A previous study showed that synthesised AgNPs using *Cleistanthus collinus* leaf extract inhibited DPPH by 43.5% at 1000 *μ*g/mL [49]. The current synthesised AgNPs showed 51.39% (AgNP-L) and 49.94% (AgNP-S) at 500 *μ*g/mL. Previous studies reported that AgNPs showed 51% of DPPH inhibition at 200 *μ*g/mL for AgNPs synthesised with *Cassia tora* leaf extract [50] and 80% inhibition at 100 *μ*g/mL for AgNPs synthesised from the leaf extract of *Croton bonplandianum* [51].

The reaction of DPPH towards antioxidants occurs through a hydrogen atom donor and electron transfer [52]. The synthesised AgNPs would be rich in hydrogen after adding the free radical (DPPH). Accordingly, the colour change from purple to yellow is a result of the conversion of free radical DPPH• (2,2-diphenyl-1-picrylhydrazyl radical) to non-free radical DPPH-H (2,2-diphenyl-1-picrylhydrazine). This is due to the transfer of hydrogen from AgNPs to free radicals in developing stable products [51]. The conjugation of biocompounds to silver ions has caused DPPH radical scavenging [53]. Therefore, biosynthesised AgNPs have potential as antioxidative agents. Although DPPH assay is simple and easy, it has its limitations. Samples that react rapidly with peroxyl radicals may either react slowly or not at all towards DPPH [52]. Therefore, the samples were further analysed using ABTS and FRAP assays.

Figure 1(b) demonstrates the antioxidant activity dependent on the ABTS radical scavenging assay. AgNPs with IC_50_ antioxidant activity of 304.31 *μ*g/mL (AgNP-L) and 326.83 *μ*g/mL (AgNP-S) are lower than CNL and CNS IC_50_ (>500 *μ*g/mL). The IC_50_ for BHA is less than 31.25 *μ*g/mL, and for C-AgNP, it is recorded at 341.81 *μ*g/mL. The ABTS radical scavenging inhibition of all tested samples shows a dose-dependent manner. The reduction of free radicals is significantly increased at higher concentrations. The results obtained, however, also show that the sample reduction of ABTS•+ is significantly lower than BHA (*p* < 0.05). Based on the data, CNL has a higher activity for each concentration and is significantly different (*p* < 0.05) from CNS. AgNP-L and AgNP-S also showed significantly different (*p* < 0.05) results at every concentration, with AgNP-L possessing higher activity of ABTS scavenging compared to AgNP-S.

The ABTS assay defines how efficient antioxidants are at scavenging ABTS and forming the ABTS radical 2,2′-azino-bis(3-ethylbenzothiazoline-6-sulphonic acid (ABTS•+). Antioxidants serve as agents for donating hydrogen. The blue/green colour of ABTS•+ is produced from the reaction of ABTS with a strong oxidising agent (potassium persulphate) which produces radical cations [54].

From the calibration curve (*y* = 0.0017*x* + 0.0451; *R*^2^ = 0.9992), the FRAP values were calculated and expressed as mM Fe(II) per *μ*g of the sample (*μ*mol/L Fe(II)/*μ*g sample). The calibration curve was determined using (FeSO_4_.7H_2_O).  Figure 1(c) shows the antioxidant activity results based on the FRAP assay. The FRAP activity of all tested samples increased in a dose-dependent manner. There was no significant difference (*p* < 0.05) between CNL and CNS. However, the difference between plant extracts and AgNPs (AgNP-L and AgNP-S) was significant (*p* < 0.05), with AgNP-L showing higher activity compared to AgNP-S. At the highest concentration of AgNPs (500 *μ*g/mL), the antioxidant activity of AgNP-L was found to be 872.389 *μ*mol/L Fe(II) and AgNP-S [612.770 *μ*mol/L Fe(II)] compared to the plant extracts with 110.445 *μ*mol/L Fe(II) (CNL) and 152.260 *μ*mol/L Fe(II) (CNS), respectively.

The FRAP assay is based on the principle of reducing antioxidants from ferric 2,4,6-tripyridyltriazine (Fe(III)-TPTZ) to ferrous (Fe(II)-TPTZ) complexes. Antioxidants act as electron donors. The colour of the end product (Fe(II)-TPTZ) is blue, and the antioxidant capacity is directly proportional to the colour intensity [55, 56].

### 3.3. Cytotoxicity Activities

Figure 2(a) shows the percentage of viability for MCF-7 after treatment with different samples. All samples showed a reduction in viable cells as the concentrations of samples increased. The IC_50_ was observed at 117.43 *μ*g/mL for AgNP-S whereas the values were more than 200 *μ*g/mL for CNL, CNS, AgNP-L, and C-AgNP. When the maximum sample concentration (200 *μ*g/mL) was used, cell viability using plant extract was higher: CNL (77.05%) and CNS (72.10%) compared to synthesised AgNPs; AgNP-L (57.24%) and AgNP-S (26.47%). AgNP-L and AgNP-S showed lower cell viability compared to C-AgNP (83.27%). All samples tested showed a significant difference from untreated cells (control) (*p* < 0.05) at 100 and 200 *μ*g/mL concentrations. Both AgNP-L and AgNP-S demonstrated a substantial difference from the control at the lowest concentration (12.5 *μ*g/mL). AgNP-S showed the lowest cell viability compared to other samples (CNL, CNS, AgNP-L, and C-AgNP).

Figure 2(b) shows the percentage viability of HT-29 after treatment. All samples showed a decrease in cell viability when the concentrations increased. The IC_50_ for AgNP-L was 78.47 *μ*g/mL, while the CNL, CNS, AgNP-S, and C-AgNP were more than 200 *μ*g/mL. The IC_50_ for 5-Fu was less than 12.5 *μ*g/mL. At the maximum concentration (200 *μ*g/mL), the viabilities of AgNP-L (22.44%) and AgNP-S (74.00%) were higher than those of the plant extracts which were CNL (73.91%) and CNS (78.82%). Both AgNP-L and AgNP-S showed lower viability compared to C-AgNP (65.61%). All the samples examined showed a significant difference (*p*< 0.05) from the control at concentrations of 50, 100, and 200 *μ*g/mL. AgNP-L displayed a higher sensitivity relative to AgNP-S as AgNP-L showed a large difference as compared to the control at the lowest concentration (12.5 *μ*g/mL).

Figure 2(c) shows the percentage of viable HeLa after treatment. The IC_50_ for AgNP-L is 175.35 *μ*g/mL while IC_50_ for CNL, CNS, AgNP-S, and C-AgNP were more than 200 *μ*g/mL and 5-Fu was less than 12.5 *μ*g/mL. At the highest concentrations of samples used (200 *μ*g/mL), the cytotoxic effects of AgNP-L (43.87%) and AgNP-S (54.33%) were higher compared to plant extracts which were CNL (87.72%) and CNS (90.23%). Both AgNP-L and AgNP-S showed higher cytotoxicity activity compared to C-AgNP (79.75%). All the samples analysed showed substantial variations at concentrations of 100 and 200 *μ*g/mL. AgNP-L demonstrated a significant difference relative to AgNP-S, which was not significant at the lowest concentration of 12.5 *μ*g/mL.

The MTS assays were used to determine the viability of the cancer cells (MCF-7, HT-29, and HeLa) after treating with samples. MTS solution is based on tetrazolium salt which measures the mitochondrial dehydrogenase activity of viable cells. The cell produces a dark purple formazan product when tetrazolium salt is cleaved by active mitochondria. Therefore, it can be used to measure the viability of the cells since the reaction only occurs in active living cells. If the cells die, they lose the ability to convert MTS into formazan [57]. The determined values are based on the formation of colours and are directly proportional to the number of cells that are viable.

Based on the findings shown, both AgNP-L and AgNP-S have produced higher cytotoxicity effects compared to plant extracts (CNL and CNS). The antiproliferative activities are categorised into four groups according to the values of IC_50_: ≤20 *μ*g/mL (active), >20–100 *μ*g/mL (moderately active), >100–1000 *μ*g/mL (weakly active), and >1000 *μ*g/mL (inactive) [58]. According to the National Cancer Institute (NCI), a crude extract is considered active for anticancer activity if it has an IC_50_ of less than 20 *μ*g/mL [59]. Thus, the AgNPs were in the group weakly active as the IC_50_ value of AgNP-L was more than 200 *μ*g/mL (MCF-7), 78.47 *μ*g/mL for HT-29, and 173.35 *μ*g/mL for HeLa. Also, the IC_50_ of AgNP-S was 117.43 *μ*g/mL (MCF-7) and more than 200 *μ*g/mL (HT-29 and HeLa). Furthermore, in previous experiments, it was discovered that AgNPs were not cytotoxic to 3T3-L1, a normal mouse embryonic fibroblast [22].

The disruption of the mitochondrial respiratory chain by AgNPs increases the production of ROS and DNA damage due to the interruption of ATP synthesis [60]. ROS are constantly being generated and eliminated in a biological system. The death of the cancer cell is hypothesised based on the excessive production of ROS (apoptosis) [61, 62]. The oxidative stress that induces apoptosis leads to the damage of cellular components in the cell [63]. Furthermore, the positive silver (Ag^+^) ion released by the dissolution of AgNPs causes cytotoxicity effects. Ag^+^ reacts with the thiol group of antioxidants such as glutathione and superoxide dismutase, thus leading to lipid peroxidation, oxidative stress, DNA damage, and cell death [64]. To conclude, the results indicate that AgNPs have cytotoxic effects against the cancer cell lines of MCF-7, HT-29, and HeLa.

## 4. Conclusions

Both Gram-positive and Gram-negative bacteria were inhibited by AgNP-L and AgNP-S, but the fungi response was negative. In addition, AgNP-L and AgNP-S showed the highest inhibition against *S. aureus* and lowest inhibition against *E. coli.* The results of these antimicrobial activities proved that AgNPs have the potential to be antimicrobial agents. In the DPPH, ABTS, and FRAP assays, AgNP-L and AgNP-S exhibited significantly greater antioxidant potency (*p* < 0.05) than plant extracts (CNL and CNS), which show promising potential for AgNPs as antioxidant agents. In the treatment of MCF-7, HT-29, and HeLa, both AgNP-L and AgNP-S demonstrated higher toxicity compared to CNL and CNS at similar concentrations. Furthermore, both AgNPs possessed a significant (*p* < 0.05) toxicity on all the cancer cells compared to the control. To conclude, the AgNPs have demonstrated potential as anticancer agents. However, more research is nseeded to support the potential for human cancer treatment. From all the studies conducted thus far, biologically synthesised AgNPs from *C. nutans* are simple and eco-friendly and have great potential to be applied as nanomedicine.

## Figures and Tables

**Figure 1:** (a) DPPH, (b) ABTS, and (c) FRAP assays. Samples with different lower case superscript letters differ significantly (*p* < 0.05) between them (mean ± SD, *n* = 3).

**Figure 2:** Cell viability after 72 h at different concentrations (12.5–200 *μ*g/mL) on (a) MCF-7, (b) HT-29, and (c) HeLa. The ^*∗*^ symbol (*p* < 0.05) represents the significant difference between the sample and control (untreated cells) (mean ± SD, *n* = 3).

**Table 1:** Inhibition zones (mm) of the biosynthesised silver nanoparticles against microorganisms using the disc diffusion method (mean ± SD, *n* = 3); mean values are significantly different (*p* < 0.05) between tested samples in each particular bacterium/fungus with different lower case superscript letters a, b, c, and d.

Samples	Inhibition zone (mm)						
	Gram-positive bacteria			Gram-negative bacteria		Fungi	
	SA	SE	SP	EC	PA	CA	CG
CNL	0.000^a^	0.000^a^	0.000^a^	0.000^a^	0.000^a^	0.000^a^	0.000^a^
CNS	0.000^a^	0.000^a^	0.000^a^	0.000^a^	0.000^a^	0.000^a^	0.000^a^
AgNP-L	11.350 ± 0.243^b^	11.597 ± 0.311^b^	10.260 ± 0.125^b^	9.220 ± 0.433^b^	10.073 ± 0.280^b^	0.000^a^	0.000^a^
AgNP-S	11.517 ± 0.519^b^	10.153 ± 0.232^c^	10.493 ± 0.345^b^	9.247 ± 0.081^b^	10.000 ± 0.305^b^	0.000^b^	0.000^a^
C-AgNP	0.000^a^	0.000^a^	0.000^a^	0.000^a^	0.000^a^	0.000^b^	0.000^a^
dH_2_O	0.000^a^	0.000^a^	0.000^a^	0.000^a^	0.000^a^	0.000^b^	0.000^a^
Gentamycin	21.957 ± 0.486^c^	25.543 ± 0.440^d^	22.967 ± 0.799^c^	21.840 ± 0.155^c^	17.530 ± 0.521^c^	ND	ND
Nystatin	ND	ND	ND	ND	ND	17.367 ± 0.136^c^	21.200 ± 0.200^b^

ND = not determined.

**Table 2:** Inhibition zones (mm) of the biosynthesised silver nanoparticles against tested microorganisms using the well diffusion method (mean ± SD, *n* = 3); mean values are significantly different (*p* < 0.05) between tested samples in each particular bacterium/fungus with different lower case superscript letters a, b, c, and d.

Samples	Zone of inhibition (mm)						
	Gram-positive bacteria			Gram-negative bacteria		Fungi	
	SA	SE	SP	EC	PA	CA	CG
CNL	0.000^a^	0.000^a^	0.000^a^	0.000^a^	0.000^a^	0.000^a^	0.000^a^
CNS	0.000^a^	0.000^a^	0.000^a^	0.000^a^	0.000^a^	0.000^a^	0.000^a^
AgNaP-L	18.290 ± 0.303^b^	16.987 ± 0.652^b^	13.913 ± 0.311^b^	12.830 ± 0.607^b^	14.160 ± 0.436^b^	0.000^a^	0.000^a^
AgNaP-S	17.237 ± 0.123^c^	17.000 ± 0.146^b^	13.730 ± 0.191^b^	13.413 ± 4.500^b^	14.140 ± 4.500^b^	0.000^a^	0.000^a^
C-AgNaPs	0.000^a^	0.000^a^	0.000^a^	0.000^a^	0.000^a^	0.000^a^	0.000^a^
Gentamycin	27.81 ± 0.206^d^	31.84 ± 0.138^c^	26.42 ± 0.678^c^	24.45 ± 0.116^c^	26.78 ± 0.102^c^	ND	ND
dH_2_O	0.000^a^	0.000^a^	0.000^a^	0.000^a^	0.000^a^	0.000^a^	0.000^a^
Nystatin	ND	ND	ND	ND	ND	26.267 ± 4.500^b^	31.285 ± 5.511^b^

ND = not determined.

**Table 3:** MIC and MBC of tested samples against microorganisms.

Samples	MIC (*μ*g/mL)					MBC (*μ*g/mL)				
	SA	SE	SP	PA	EC	SA	SE	SP	PA	EC
AgNP-L	250	250	250	250	125	250	250	250	250	125
AgNP-S	250	250	250	125	125	250	250	250	125	125
Gentamicin	31.25	62.5	31.25	62.5	125	31.25	31.25	31.25	62.5	125

## Data Availability

The data used to support the findings of this study are included within the article.
